# Influence of Compression Thresholds and Maximum Power Output on Speech Understanding with Bone-Anchored Hearing Systems

**DOI:** 10.1155/2021/1518385

**Published:** 2021-10-22

**Authors:** Tom Gawliczek, Wilhelm Wimmer, Marco Caversaccio, Martin Kompis

**Affiliations:** ^1^Department of ENT, Head and Neck Surgery, Inselspital Bern, University of Bern, 3010 Bern, Switzerland; ^2^Hearing Research Laboratory, ARTORG Center for Biomedical Engineering Research, University of Bern, Bern 3008, Switzerland

## Abstract

Bone-anchored hearing systems (BAHS) transmit sound via osseointegrated implants behind the ear. They are used to treat patients with conductive or mixed hearing loss, but speech understanding may be limited especially in users with substantial additional cochlear hearing losses. In recent years, BAHS with higher maximum power output (MPO) and more advanced digital processing including loudness compression have become available. These features may be useful to increase speech understanding in users with mixed hearing loss. We have tested the effect of 4 combinations of two different MPO levels (highest level available and level reduced by 12 dB) and two different compression thresholds (CT) levels (50 dB and 65 dB sound pressure level) in 12 adult BAHS users on speech understanding in quiet and in noise. We have found that speech understanding *in quiet* was not influenced significantly by any of the changes in these two fitting parameters. In contrast, in users with average bone-conduction (BC) threshold of 25 dB or more, speech understanding *in noise* was improved by +0.8 dB to +1.1 dB (*p* < 0.03) when using the higher MPO level. In this user group, there may be an additional, but very small benefit of +0.1 dB to +0.4 dB when using the lower rather than the higher CT value, but the difference was not statistically significant (*p* > 0.27). In users with better average BC thresholds than 25 dB, none of the improvement was statistically significant. Higher MPOs and possibly, to a lesser degree, lower CTs seem to be able to improve speech understanding in noise in users with higher BC thresholds, but even their combined effect seems to be limited.

## 1. Introduction

For over 4 decades, bone-anchored hearing systems (BAHS) have been used successfully to treat conductive and mixed hearing loss, especially in cases where conventional hearing aids cannot be used or where they are not effective [1, 2]. BAHS consist of a retroauricularly implanted titanium screw with a skin-penetrating abutment, onto which an external sound processor with microphones, signal processing unit, and a transducer (vibrator) is mounted. Unlike conventional hearing aids, BAHS use the bone conduction (BC) path and not the air conduction (AC) path via the external ear canal to reach the inner ear.

For the first decades of their existence, the technology of BAHS did not allow for sophisticated fine tuning. Modern BAHS systems use digital signal processing and a considerable number of parameters, such as MPO and gain settings in different frequency bands have become accessible to the audiologist and have opened new possibilities for fine tuning. It was shown that meeting adequate prescriptive targets can improve speech understanding [3, 4]. On the other hand, some studies showed only small improvements in terms of speech understanding when trying to optimize fitting parameters of BAHS [5, 6].

One important limit to a wider application of BAHS is low speech understanding in users with a mixed hearing loss, especially if the sensorineural component is substantial, i.e., above approximately 25-40 dB HL. As the maximum power output (MPO) levels of BAHS are inherently and substantially lower than those of conventional hearing aids, the dynamic range, i.e., the difference between the bone conduction threshold of the user and the MPO of the BAHS can become very narrow and may limit speech understanding considerably. Fortunately, BAHS with higher MPOs (often called power devices or, more recently, superpower devices) have started to provide better preconditions for these difficult fittings. Nevertheless, the increase in speech understanding reached in this way is still limited [6].

Dynamic range compression has been shown repeatedly to improve speech understanding in users of air conduction hearing aids [7–9]. However, the fitting of hearing devices for hearing losses with a conductive component is known to differ from the fitting of purely sensorineural hearing losses [10]. Furthermore, loudness growth has been shown to differ between the AC pathway used in conventional hearing aids and the BC pathway used by BAHS [11, 12]. Therefore, it seems reasonable to assume that optimal loudness compression parameters may differ between BAHS for mixed hearing losses and AC hearing aids for sensorineural hearing losses.

The rationale behind our study was that optimizing loudness compression parameters of BAHS might improve speech understanding in everyday life. Specifically, we wanted to test the hypothesis that choosing lower compression thresholds (CT; i.e., the input level at which the loudness compression sets in) might improve speech understanding of BAHS users. We are not aware of any other studies looking into this effect, and we aimed to start to close this gap.

Because compression sets in already at lower input levels with lower CT-levels, they help to expand the dynamic range of the incoming acoustic signal, which is ultimately available at the inner ears of the users. We hypothesized that this might lead to better speech understanding, as dynamic ranges are generally narrow in fittings with BAHS, when compared to air conduction hearing aids [6, 13] and may therefore be a limiting factor. The dynamic ranges become even narrower in BAHS users with poor BC thresholds, as often seen in older persons, and in smaller devices with lower MPOs [6, 14]. For this reason, these two factors (BC thresholds and MPO levels) have been explicitly included in our study design and analysis.

## 2. Material and Methods

### 2.1. Ethics

The study was approved by the local ethical committee of Bern (KEK-BE 2018-01521) and carried out in accordance with the Declaration of Helsinki.

### 2.2. Study Population

Twelve regular BAHS users participated in the study after giving their written informed consent. Four of the volunteers were female, and 8 were male. Their ages ranged from 36 to 79 years (mean 63 years). All were German speaking, and all had a bilateral conductive hearing loss with an additional sensorineural hearing loss. Their average AC pure tone thresholds in the frequency range 500-4000 Hz (PTA_4_) were 29 to 110 (mean 78) dB HL for the side tested with the BAHS and 28 to 103 (mean 59) dB HL for the contralateral side. BC thresholds were 5 to 71 (mean 36) dB HL on the BAHS side and 5 to 50 (mean 29) dB HL for the contralateral side. For data analysis and visual representation in the figures, we use the BC thresholds of the ear with the better BC threshold, as this threshold correlates better with the aided outcome with BAHS than that of the ipsilateral ear [15, 16].

### 2.3. Speech Processor and Settings

Testing was carried out with a Baha 5 SuperPower audio processor (Cochlear Inc. Mölnlycke, Sweden). The processor was fitted individually for each participant using BC-direct threshold measurements. Automatic sound classification, position compensation, microphone directionality, and noise reduction were deactivated.

Four different combinations of settings of the parameters were programmed for each volunteer. MPO was either maintained at the highest level possible by the hardware of the processor used (“High MPO”) or reduced by 12 dB over the entire frequency range (“Low MPO”). These MPO settings are shown in Figure 1. The lower level corresponds approximately to the MPO levels of a medium-power BAHS processor [17]. Compression thresholds were set either to 50 dB SPL (“CT 50 dB”) or to 65 dB (“CT 65 dB”). The compression ratio above these levels was 2.5. This value was chosen as it is, along with the higher of the two CT levels tested (65 dB SPL), the default setting of the most recently introduced bone conduction system by the same manufacturer [18]. The other CT levels was chosen to be 50 dB SPL, as it is considerably lower than the first CT level, thus increasing the probability to find effects on speech intelligibility, while both CT values are still in a reasonable range used for hearing aid fittings [7, 9, 19].

After an initial pure tone audiometry (AC and BC thresholds), all measurements were performed with a single audio processor mounted on the abutment of each subject. In those 3 participants, who had bilateral implants, the side with the better BC thresholds was chosen for all tests. During the measurements, the ear contralateral to the BAHS was plugged (E.A.R. classic II, 3 M Inc., Berkshire, UK) in all subjects with the exception of 3 participants, who had a complete atresia of the external auditory canal.

Figure 1 shows a representation of the BC thresholds of all 12 subjects along with the two MPO level settings converted to dB HL [20].

### 2.4. Setup and Testing

All measurements took place in a soundproof chamber (6.0 × 4.1 × 2.2 m^3^) with an average reverberation time of 0.14 s. Four JBL Professional ControlVR 1 PRO loudspeakers (JBL Professional, Northridge, California, USA) were placed to the left, right, front, and rear of the listener at a distance of 1 m. This setting was identical to that used in a previous study [6].

Speech understanding was measured in quiet and in noise for each subject and for each combination of the 2 MPO levels and 2 CT levels described above. The order of the measurements was changed systematically between subjects to minimize the influence of learning or fatigue. Speech reception thresholds levels in quiet were assessed using 2-digit German numbers. The presentation level required for 50% speech understanding was recorded. Word understanding in quiet was measured with lists of 20 German monosyllabic words from the Swiss version of the Freiburg test [21], presented at 65 dB SPL from the front loudspeaker.

Speech reception thresholds in noise were measured using the adaptive German matrix test [22]. Lists of 30 test sentences were presented from the front loudspeaker, and 4 uncorrelated instances of speech babble noise with the same long-term spectrum of the test sentences were played continuously from all 4 loudspeakers [23] at a resulting total level of 65 dB SPL.

### 2.5. Data Analysis

For the statistical analysis mixed-effect linear models were used. Test conditions (MPO level and CT level) were defined as fixed effects. For the post hoc analyses in Table 1, a general linear hypothesis testing using two-tailed tests and Holm correction for multiple testing was used. The statistical environment ‘R' was used for all calculations (R Core Team 2021, version 4.0.5, with packages ‘lme4' version 1.1-26, and ‘multcomp' version 1.4-17).

Sample size was calculated for speech understanding in noise. As the standard deviation is below 1 dB [22], a small, but still useful improvement of 1 dB in signal-to-noise ratio can be expected to be found with 12 subject (significance level *p* = 0.05, power 80%).

In Figure 2 (word recognition scores quiet), where the range of the results on the *y*-axis is limited to 0-100%), fitted Sigmoid curves are shown. For speech reception thresholds in quiet and in noise, where there is no such theoretical upper limit for the values on the *x*-axis, second-order polynomial functions were used.

For a part of the analysis, the study population was divided into 2 subgroups. Subgroup A included all participants with a mean PTA_4_ BC threshold (average between the values at 0.5, 1, 2, and 4 kHz) between 0 and 25 dB (*N* = 6) and group B between 25 and 50 dB (*N* = 6).

## 3. Results

Figure 3 shows aided speech reception thresholds (SRT) in quiet as a function of the sensorineural hearing loss (average BC threshold at the frequencies 0.5, 1, 2, and 4 kHz). SRTs increase with increasing BC thresholds. The difference between group A (mean 34 dB) and group B (mean 45 dB) is statistically significant (*p* < 0.001). However, there are no significant differences between the SRTs when using the higher or lower MPO or CT level (degrees of freedom dF = 33, *t* < 1.204, *p* > 0.237) and all fitted curves run close together.

Figure 2 shows a similar representation for the monosyllabic word recognition scores. Scores drop from an average of 98% in group A to 75% in group B (*p* < 0.001). Again, different MPO and CT levels have no significant (dF = 33, *t* < 0.242, *p* > 0.81) impact on speech understanding and the 4 fitted curves lie close together.

Figure 4 shows the corresponding representation for the speech reception thresholds in noise. Similar to the measurements in quiet, SRTs in noise become worse for higher bone conduction hearing thresholds. Their average is -6.5 dB for group A and -3.5 dB for group B (*p* < 0.001). In contrast to the measurements in quiet, the fitted curves for the 4 different test conditions are now somewhat further apart and statistically significant differences emerge, as shown in Table 1.

An increase of the MPO level by 12 dB improves speech understanding in noise in group B significantly by +0.8 at CT = 65 dB to +1.1 dB at CT = 50 dB. No other change in the fitting parameters under investigation causes an improvement that reaches statistical significance. The impact of a higher MPO is smaller for group A than for group B. While there is no statistically significant effect of lowering the compression threshold from 65 dB to 50 dB, it does improve SRTs in noise in both groups and for both MPO levels by +0.1 to +0.7 dB on average. As a result, the combination of the higher MPO level and the lower CT level give the best average SRTs in both groups.

## 4. Discussion

Our results show that choosing a higher MPO in BAHS users with a mixed hearing loss and a sensorineural component of more than approximately 25 dB HL can improve speech understanding in noise significantly, but modestly by approximately 1 dB in signal-to-noise ratio (SNR). The benefit for users with a less pronounced sensorineural component is smaller and does not reach statistical significance in our study group. These results are comparable to those of an earlier study using BAHS and different MPOs [6]. They are better (i.e., we found larger improvements) when compared to another study, in which the difference between the 2 MPOs which were compared was only 5 dB, as opposed to 12 dB in our study.

As to compression thresholds (CT), our rationale was that a lower CT might lead to better speech understanding as a widened range of the acoustic input levels could be mapped on the dynamic range of the BAHS users. This range may be rather narrow, being limited by their BC thresholds at one end and the MPO of their BAHS at the other end. Indeed, as Table 1 shows, speech understanding in noise is improved in both subgroups and for both MPO levels tested, but the average improvements of +0.1 to +0.7 dB in SNR are small and do not reach statistical significance. Overall, the combination of a low CT and high MPO improves SNR by 0.7 dB in group A and by 1.2 dB in group B. While we did not find a proof that lower CTs are significantly better for BAHS users in terms of improved speech understanding, the notion should not be discarded entirely either. Further research with a larger range of CTs, more subjects and possibly combined with a range of different compression ratios might show more definitive and more promising results. We are not aware of any studies, which would allow a direct comparison with our results. Kurz et al. [5] tested different compression ratios—but not different compression thresholds—and found no statistically significant effects. A review by McCreery et al. [9] shows evidence for the benefit of wide dynamic range compression with low CTs in air conduction hearing aids, but the comparison between studies with different CTs remains difficult.

For speech understanding in quiet, no effect of the choice of different MPO or CT levels was found. One reason for this finding may be that speech in quiet is generally easier to understand and distortions caused, e.g., by too narrow dynamic ranges are less detrimental, when only a single target signal is present, and not a mix of speech and noise. Finding no significant effect on speech understanding in quiet is rather typical for several types of studies involving BAHS and individual fitting parameters, such as MPO or compression ratio [5, 6] or even the comparison of different sound processors (e.g., [24, 25]).

In contrast, considerable improvements in speech understanding with BAHS by improving their fitting have been found by Hodgetts et al. [3]. In their work, a number of parameters including the frequency responses were changed simultaneously to fit a prescription target. In contrast, changing only single fitting parameters such as MPO, CT, or the compression ratio seems to yield only modest improvements as shown in the present study and in earlier investigations [5, 6]. Nevertheless, such studies could provide valid guidelines in clinical routine when choosing a value for a fitting parameter in a given BAHS user. Furthermore, the small benefits may be additive, as suggested with the combination of higher MPOs and lower CTs in this study.

## 5. Conclusions

Higher MPO levels lead to increased speech understanding in noise in BAHS users with BC thresholds above approximately 25 dB. The improvement is in the order of magnitude of 1 dB in SNR for an increase of 12 dB in MPO. No significant effect on speech understanding in quiet or in users with better BC-thresholds was found. Lowering compression thresholds from 65 dB to 50 dB may increase speech understanding in noise additionally by small amounts of +0.1 to +0.7 dB in SNR, but statistical significance was not reached in any condition in our study. For BAHS fitting, it may be beneficial to choose devices with high MPOs when treating patients with poor BC thresholds (approximately 25 dB or more) and using lower rather than higher compression threshold may give a small additional advantage.

## Figures and Tables

**Figure 1:** (a) BC hearing thresholds of the better ears of the 12 study subjects (solid line denotes mean). (b) The two maximum power output (MPO) levels compared in the study, converted to dB HL for easier comparison.

**Figure 2:** Word recognition scores (monosyllabic words) in quiet as a function of the average BC threshold (0.5-4 kHz). Individual data points and fitted curves (sigmoid) are shown for the 4 test conditions.

**Figure 3:** Aided speech reception thresholds (SRT) in quiet as a function of the average BC threshold of the participants (pure tone average PTA_4_ over the frequencies 0.5, 1, 2, and 4 kHz). Individual data points and 2^nd^-order polynomial fits are shown for each of the 4 test conditions.

**Figure 4:** Speech reception thresholds (SRT) in noise as a function of the average BC threshold (0.5-4 kHz). Individual data points and fitted curves (2^nd^-order polynomial) are shown for each test condition.

**Table 1:** Mean improvement of speech reception thresholds in noise, when keeping one fitting parameters constant and changing the other one.

Fixed parameter	Changed parameter	Group A (average BC threshold 0-25 dB)	Group B (average BC threshold 25-50 dB)
CT = 50 dB	MPO low ➔ high	+0.5 dB (*p* = 0.33) ^ns^	+1.1 dB (*p* = 0.007) ^∗∗^
CT = 65 dB	MPO low ➔ high	+0.0 dB (*p* = 0.98) ^ns^	+0.8 dB (*p* = 0.03) ^∗^
MPO = high	CT 65 dB ➔ 50 dB	+0.7 dB (*p* = 0.16) ^ns^	+0.4 dB (*p* = 0.27) ^ns^
MPO = low	CT 65 dB ➔ 50 dB	+0.3 dB (*p* = 0.62) ^ns^	+0.1 dB (*p* = 0.69) ^ns^

ns: not significant.

## Data Availability

The data used to support the findings of this study are available from the corresponding author upon request.

## Abbreviations

AC: Air conduction
BAHS: Bone-anchored hearing system
BC: Bone conduction
CT: Compression threshold
MPO: Maximum power output
n.s.: Not significant
PTA_4_: Pure tone average thresholds at 0.5, 1, 2, and 4 kHz.
